# Unani Formulation Habb-e-Suranjan: A Treasure of Biological Activities

This article has been retracted.

**DOI:** 10.1155/2022/1640193

**Published:** 2022-07-26

**Authors:** Ansari Imtiyaz Ahmed Tufail Ahemad, Qazi Majaz Ahamad Aejazuddin, G. J. Khan, Abdulrhman Alsayari, Shadma Wahab, Sharuk L. Khan, Noor Jahan Akter, Md. Rezaul Islam, Arpita Roy, Fahadul Islam

**Affiliations:** ^1^J.I.I.U's Ali-Allana College of Pharmacy, Akkalkuwa, Nandurbar, Maharashtra 425415, India; ^2^Department of Pharmacognosy, College of Pharmacy, King Khalid University, Abha 61421, Saudi Arabia; ^3^Complementary and Alternative Medicine Unit, College of Pharmacy, King Khalid University, Saudi Arabia; ^4^MUP's College of Pharmacy (B Pharm), Degaon, Risod, Washim, Maharashtra 444504, India; ^5^Department of Pharmacy, Faculty of Allied Health Sciences, Daffodil International University, Dhaka 1207, Bangladesh; ^6^Department of Biotechnology, School of Engineering & Technology, Sharda University, Greater Noida, India

## Abstract

Habb-e-Suranjan (HES), an Unani formulation, has been studied for its anti-inflammatory properties in both *in vitro* and *in vivo* experiments. HES is recommended for arthritis, gout, and joint pain. The current endeavor is an attempt to put it to the test and verify its efficacy scientifically. It was tested for DPPH, hydroxyl, and nitric oxide scavenging activities. It was shown that HES had the greatest TAC and FRAC values when compared to catechin and ascorbic acid. HES exhibited DPPH and hydroxyl radical scavenging activity that was dose-dependent. Incubation of sodium nitroprusside solutions in PBS at 25°C for 150 min resulted in the production of nitric oxide. Nitric oxide production was effectively decreased by HES. Anti-inflammatory medications boosted the migration of PMN cells toward the chemoattractant FMLP in an agarose experiment of PMN chemotaxis. In carrageenan-induced rat paw edema, in the HES-treated group, paw thickness was 3.021 ± 0.084 at *t* = 0, but it showed an increase in paw inflammation after one hour, i.e., 3.195 ± 0.082 cm which again showed a decrease in paw thickness up to 4th hour, i.e., 3.018 ± 0.078, 2.98 ± 0.032, and 2.684 ± 0.061 at *t* = 2, 3, and 4, respectively. It showed again getting back to the normal thickness of paw at *t* = 24 hrs, i.e., 3.029 ± 0.118 cm. It is concluded that the formulation is potent enough and can be used effectively for the treatment of inflammation and associated health issues. Moreover, there is much scope to evaluate its effectiveness using different *in vitro* and *in vivo* models.

## 1. Introduction

Unani System of Medicine is Graeco-Arabic medicine founded by Hippocrates and Galen and refined by Arabian and Persian doctors such as Rhazes (al Razi) and Avicenna (Ibn-e-Sina), Al-Zahrawi, and Ibn Nafis throughout the Middle Ages. Buqrat (460-377 BC), also known as Hippocrates, was a descendant of Aesculapius and is regarded as the “Father of Unani Medicine” [1, 2]. It began around 2500 years ago in Greece, and it has been employing drugs that are 90% herbal, 4-5 percent animal, and 5-6 percent mineral in nature. It is not only the original science of medicine but also a vast repository of medical ideas and philosophies that can be extremely beneficial to both medicine and science in general. Diseases are thought to disrupt the body's normal temperament and humor equilibrium. So regimental therapy (Ilaj Bil-Tadabeer) and pharmacology (Ilaj Bil-Dawa) have been used since ancient times with the express purpose of restoring humor equilibrium and correcting aberrant temperament. When this method of treatment fails, surgery (Ilaj Bil-yad) is recommended as a last resort [3, 4].

Many researchers are working on herbal medicine to prove its effectiveness in a variety of diseases including COVID-19 [5–14]. It is well documented that herbal medicine has proven its role in the treatment of inflammation, obesity, cancer, diabetes mellitus, etc. [15–19]. Although it is thought that the usage of herbal remedies dates back to 1550 BC in Egypt, many of its pharmacological effects are still unknown. Only approximately a quarter of the estimated 800,000 plant species on the planet have been classified, and only a small percentage of these have been tested for pharmacological efficacy. More plant-based drugs were sought to aid in the treatment of the various ailments that still afflict society [20–23].

For the promotion and maintenance of health, the Unani system of medicine places a strong focus on lifestyle management. Diet, lifestyle, emotions, interactions with the environment, and even spiritual considerations are all taken into account [24]. It takes into account both external elements such as seasons, air quality, food and beverages, and internal aspects such as sleep and wakefulness, movement and rest, evacuation and retention, and so on. The Unani system of medicine is extremely relevant to modern healthcare because of its ability to promote health and disease prevention through nondrug lifestyle variables [7, 25].

Elwa/Sibr (*Aloe barbadensis*), Halela (*Terminalia chebula*), and Suranjan (*Colchicum luteum*) were combined in equal amounts in the test formulation, Habb-e-Suranjan (HES), which was made under the supervision of a GMP-certified pharmacist at CRIUM, Hyderabad, and sent to the research site. Three times a day, patients were instructed to apply 5 ml of lukewarm oil to the afflicted joints in the morning and evening twice a day for two weeks after taking HES (500 mg each) for two weeks [26].

Subchronic oral toxicity studies of HES in albino Wistar rats were investigated by Ghazanfar et al. [3]. The antiarthritic impact of Unani pharmacopoeial formulations of HES and Raughan-e-Suranjan in Waja-al-Mafasil was researched and assessed by Ahmed et al. [26]. Suhail et al. [27] studied and explained Habb/pill (plural: Huboob) is a solid medicinal preparation, made by mixing powdered drugs in a suitable binder (water/oil/resin of plant) and made into a round and uniformly shaped balls of the required size. Habb-e-Suranjan is one of the common Huboob or pills used in the Unani system of medicine from ancient times. This polyherbal formulation is being used as an analgesic for the treatment of various types of joint disorders and nerve pains like Waja'-al-Mafaasil (Arthralgia), Waja'-al-A'saab (Neuralgia), Irq-al-Nasa (Sciatica), and Niqris (Gout). It is also used in Qabz (constipation). A comparative study of the therapy of primary gout with HES and allopurinol was conducted by Akhtar and Siddiqi [28]. HES contains different potential ingredients such as Elwa (Musabbar)-Aloe vera (Indian Aloe) extract (11.29%), Tuhkm Soya (11.29%), Turbud Safed (Turpeth)-Ipomoea Turpethum (30.64%), Habb-ul-Neel-Indigo (11.29%), Suranjan Shirin (Colchicum Corm)-Colchicum Luteum (25.80%), Guggulu-Gum Guggul-Commiphora Mukul (4.83%), and Mastagi-Mastiche (4.83%) [29].

A review of the literature revealed that the *in vivo* and *in vitro* anti-inflammatory potential activity of Unani formulation HES was not previously conducted to evaluate the formulation's traditional claim as anti-inflammatory and antioxidant. Therefore, present work was aimed at performing phytochemical screening and *in vivo* as well as *in vitro* anti-inflammatory activities of HES.

## 2. Material and Methods

### 2.1. Drugs and Chemicals Used

Habb-e-Suranjan (HES) was purchased from the local Unani medical store of Nandurbar, Maharashtra, India. Oxycodone (Sigma-Aldrich, St. Louis, MO, USA) and 0.9% sodium chloride (Hospira, Lake Forest, IL, USA), Folin-Ciocalteu reagent, 2,2-diphenyl-1-picryl hydroxyl radical (DPPH), phenazine methosulfate, nicotinamide adenine dinucleotide, sodium nitroprusside (SNP), trichloroacetic acid (TCA), thiobarbituric acid (TBA), and L-ascorbic acid were purchased and procured from Lab Trading Laboratory, Aurangabad. Catechin and rutin were purchased from Sigma Chemicals, India.

### 2.2. Physicochemical Analysis and Preliminary Phytochemical Screening of Habb-e-Suranjan

The specification of the HES mixture was evaluated by performing physicochemical analyses such as appearance, color, taste, odor, pH value, friability, hardness, weight change, and disintegration time. Initial phytochemical testing of the powder of HES tablets was carried out following previously documented procedures [12].

### 2.3. Animals Used and Ethical Approvals

36 male Wister rats and 30 male mice weighing about 150-200 g and 25-30 g each were used for the study. They were fed with a standard pellet diet and were supplied with water ad libitum, housed less than 12 h light/dark cycles, with controlled temperature (22-25°C). At least one week before the trial began, the animals were acclimated to the new environment. Care of the animals and experimental procedures were done according to the guidelines of the Institutional Animal Ethics Committee (IAEC) having approval number CPCSEA/IAEC/JLS/16/07/21/11.

### 2.4. *In Vivo* Anti-inflammatory Activity

#### 2.4.1. Carrageenan-Induced Rat Paw Edema

The carrageenan-induced rat paw edema method was used to test the anti-inflammatory properties of HES. The 24 rats were split up into four equal groups, each with six rats. Group 1 (control group) was injected with saline and provided with the vehicle, group 2 (carrageenan control) was injected with carrageenan and was orally treated with the vehicle, group 3 (treatment 1) was treated with HES 100 mg/kg p.o., and group 4 (standard group) was treated with diclofenac sodium 100 mg/kg. Carrageenan, a substance that causes inflammation, and the conventional and experimental medications were all given intravenously via the use of sterile saline water.

This research began by treating the animals with the medications stated above (vehicle, standard, and three treatments). Carrageenan solution was injected into the subplantar area of the right hind paw one hour after the previous treatment to produce edema. Carrageenan injections increased the thickness of the paws, indicating edema. After carrageenan injection, measurements were taken at 0, 1, 2, 3, 4, and 24 hrs using the Plethysmometer. The difference between the paw thickness at “0 hour” and the paw thickness at the corresponding hours was used to calculate the increase in paw thickness [30, 31].

#### 2.4.2. Paw Withdrawal Threshold (Von Frey Test)

Mechanical allodynia: the rat was placed individually on an acrylic cage elevated maze and adopted for the test environment for a minimum of 15 min. Von Frey filament was attached to the rat's plantar aspect of the hind paw from the mesh floor's base. When enough filament force was given to the paw, it bent slightly and held there for a brief period. Withdrawal of the paws was seen as a favorable reaction. Oxycodone was used as a standard drug; it was given at a dosage of 150 g/0.1 ml/kg after being dissolved in 0.9 percent sodium chloride [32, 33].

#### 2.4.3. Acetic Acid-Induced Vascular Permeability

Both HES and diclofenac were given to rats at doses of 100 mg/kg intravenously, and the vehicle was used as a control. 2 percent Evan's blue solution was administered i.v. into the tail vein of each rat 1 hour after the treatments. A solution of 6.5% acetic acid (in saline) was administered i.p. into each mouse 10 minutes later at a dose of 10 ml/kg body weight into each animal. The rats were euthanized and their peritoneal cavity was cleaned three times with saline (10 ml) after 30 minutes of acetic acid administration. The saline washes were centrifuged at 3500 rpm for five minutes. A plate reader was used to measure the absorbance at 590 nm of the collected supernatant. In micrograms, Evan's blue extravasation was counted using a standard curve [34, 35].

#### 2.4.4. Tail Immersion Test

Rats were divided into 6 animals in each group. The lower part of the tail (5 cm) was immersed in a beaker containing water maintained at 55 ± 0.5°C. The time taken for the withdrawal of the tail from the water was recorded as a reaction time, with 10 sec as a cut-off time. The reaction time was noted one hour before the administration of drugs and as well one hour after the administration. The control group was provided with saline, whereas the treatment groups were provided with HES (100 mg/kg) p.o, and dextropropoxyphene (65 mg/kg) was administered as a standard drug subcutaneously, 30 min before the test [36].

#### 2.4.5. Adjuvant-Induced Arthritis (AIA) in Rats

A kind of arthritis was induced in rats after they were injected with Freund's complete adjuvant (CFA). On day 0, rats were anesthetized with an 80 : 10 mg/kg i.p. ketamine and xylazine mixture before being injected intradermally with 0.1 ml CFA 1 mg/ml heat-inactivated Mycobacterium tuberculosis in 85 percent paraffin oil and 15 percent mannide monooleate at the tail base. Animals in the control group received a saline injection with the same volume as the experimental group rats. Grouping was done as follows: control (no adjuvant, saline), AIA (adjuvant, no treatment), HES (adjuvant, 100 mg/kg HES), and 0.1 mg/kg methotrexate (MTX); it is the most utilized antirheumatic drug and hence was used as a standard drug administered p.o. The injections were administered every day for 27 days [37]. Blood was drawn from the retroorbital plexus to conduct laboratory testing on hematological parameters. Red blood cell (RBC), white blood cell (WBC), platelet count, and erythrocyte sedimentation rate (ESR) are among the hematological characteristics measured [38].

### 2.5. *In Vitro* Anti-inflammatory Activity

#### 2.5.1. Determination of Total Antioxidant Capacity (TAC)

Rahman et al. [39] presented a technique for determining sample TAC. This test is primarily dependent on the drugs/samples reducing Mo (VI) to Mo (V), resulting in the development of a green-colored phosphate/Mo (V) complex at acidic pH. 3 ml of a mixture comprising 0.6 M sulphuric acid, 28 mM sodium phosphate, and 1 percent ammonium molybdate was combined with 0.5 ml of samples/standards at varied concentrations of 12.5-150 *μ*g/ml. The reaction was completed by incubating the test tubes containing the above mixtures at 95°C for 10 minutes. After allowing the reaction mixture to cool to ambient temperature, the absorbance at 695 nm was measured using a spectrophotometer using a blank solution as a control. Catechin was utilized as a point of comparison. A blank solution was prepared using 3 ml of the reaction mixture, and the same amount of solvent as was used for the samples and standard. The blank was also incubated for 10 minutes at 95°C before being measured at 695 nm. Absorbance increases indicate a higher total antioxidant capacity. For each antioxidant assay, standard/samples were used at five different concentrations ranging from 12.5 to 150 *μ*g/ml. Several different concentrations were tested to see which one best reflected the reasonable rise in antioxidant activity as the concentration of the sample rose.

#### 2.5.2. Ferrous Reducing Antioxidant Capacity Assay (FRAC)

The FRAC of samples was determined using Rahman et al.'s technique [39]. The development of Perl's Prussian blue at 700 nm may be used to monitor Fe^2+^. The test tubes were filled with 0.25 ml of standard/sample solutions ranging from 12.5 to 150 g/ml, 0.625 ml of potassium buffer (0.2 M), and 0.625 ml of 1 percent potassium ferricyanide solution. It took around 20 minutes of incubation at 50 degrees Celsius to complete the reaction. The test tubes were then filled with 0.625 ml of a 10% trichloroacetic acid solution. The aforesaid combination was centrifuged for 10 minutes at 3000 rpm, after which 1.8 ml of the supernatant was removed from the test tubes and mixed with 1.8 ml of distilled water and 0.36 ml of 0.1 percent ferric chloride solution. The absorbance at 700 nm was measured using a spectrophotometer, and the results were compared to a blank. The absorbance of a blank solution containing the same reaction mixture but without the sample/standard was measured at 700 nm after incubation under the same circumstances. Higher reaction mixture absorption indicates a greater capacity to reduce. At each concentration, the experiment was performed three times.

#### 2.5.3. Radical Scavenging Activity

*(1) DPPH Radical Scavenging Assay*. The compounds' capacity to scavenge free radicals was assessed using the DPPH radical scavenging assay, as reported by Rahman et al. [39]. The capacity of the compounds to donate hydrogen atoms was assessed by decolorizing a methanol solution of 2,2-diphenyl-1-picrylhydrazyl (DPPH). In methanol solution, DPPH produces a purple/violet hue that fades to shades of yellow in the presence of antioxidants. A 0.1 mM DPPH in methanol solution was produced, and 2.4 ml of it was combined with 1.6 ml of extract in methanol at concentrations ranging from 12.5 to 150 *μ*g/ml. The solution combination was completely mixed before being stored in the dark at room temperature for 30 minutes. At 517 nm, the absorbance was determined spectrophotometrically. As a control, butylated hydroxytoluene (BHT) was utilized. The percentage of DPPH radical scavenging activity was determined by this equation: %DPPH radical scavenging activity = [(*A*_0_ − *A*_1_)/*A*_0_] × 100.

Here, *A*_0_ is the absorbance of the control, whereas the drug's/absorbance standard is *A*_1_. The IC_50_ was then determined by plotting the percentage of inhibition versus the concentration. At each concentration, the experiment was carried out three times.

*(2) Hydroxyl Radical Scavenging Activity*. By using the technique of Rahman et al., the hydroxyl radical scavenging activity of the medicines was determined [39]. This system created hydroxyl radicals by combining Fe^3+^-ascorbate-EDTA-H_2_O_2_ (Fenton reaction). In this test, the 2-deoxy-D-ribose breakdown product, which generates a chromogen when heated with TBA at low pH, is quantified. For this experiment, the reaction mixture comprised the following components: 50 mmol l^−1^ of phosphate buffer solution, 12.5-150 *μ*g/ml of drug/standard, 10.0-40.0 mol l^−1^ of sodium azide, 10.0-10.0 mg/ml of sodium deoxycholate, and 20.0-20.0 mg/ml of 2-deoxy-D-ribose (28 mmol l^−1^). At 370 degrees Fahrenheit, the mixtures were held in a water bath and the reaction was initiated by adding 0.2 ml of ascorbic acid, H_2_O_2_ (2 mmol l^−1^), and AA (2 mmol l^−1^) (10 mmol l^−1^). 1.5 ml of HCl is added after 1 hour of incubation at 370°C. For 15 minutes, the reaction mixture was heated to 100°C and then cooled with a stream of cold water. The solution's absorbance was measured at 532 nm. With the suppression of the percentage of 2-deoxy-D-ribose oxidation on hydroxyl radicals, the scavenging capability of hydroxyl radicals was determined. The proportion of hydroxyl radical scavenging activity may be calculated using the following equation: %hydroxyl radical scavenging activity = [*A*_0_ − (*A*_1_ − *A*_2_)] × 100/A_0_.

In the equation, *A*_0_ is the control's absorbance without a sample present. Sample and 2-deoxy-D-ribose were added to *A*_1_ and the absorbance was measured. When 2-deoxy-D-ribose is omitted from the sample, its absorbance is equal to *A*_2_. The IC_50_ was then determined by plotting the percentage of inhibition versus the concentration. At each concentration, the experiment was carried out three times.

*(3) In Vitro Activity of HES on Human PMN Cell*. Samples of fresh, anticoagulated blood taken from healthy human volunteers were used to isolate PMN cells. In order to extract PMN cells, 5 ml of blood was combined with 1.75 percent Dextran T-500 solution in saline and placed for 45 minutes at room temperature for sedimentation. The remaining RBCs were washed three times with PBS before being suspended in a 10% fetal bovine serum-containing RPMI-1640 medium, which was then centrifuged. The PMN cell density was set using RPMI-1640 media containing 10% fetal calf serum. As part of the in vitro testing, dilutions of the active ingredients in each of the assays were made in RPMI-1640 medium by adding 10 *μ*l of the dilution to 990 *μ*l medium. Effect on the chemotaxis of PMN cells/human PMN cell chemotaxis produced by formyl-N-methyl-leucyl-phenylalanine (FMLP) was studied in vitro using the chemotaxis test technique under agarose. The agarose solution (1.2 *w*/*v*) was prepared in Eagle's minimal essential medium (MEM) and heated to 56°C. The microscopic slides (50 × 75 mm) were produced by putting 6.0 cc of the aforementioned solution over each slide and allowing this to settle at room temperature. The slides were kept at 2-8°C for six hours. After that, 5 mm diameter wells were drilled into the settled gel, each one 4 mm in diameter. The wells were added with 20 *μ*l FMLP solution in RMPI-1640 medium whose concentration was 1 × 10^−8^ for determining the chemotaxis in response to FMLP. The surrounding wells contained 10 *μ*l PMN (1 × 10^8^ cells/ml in minimum essential medium) and 10 *μ*l of each drug solution. The slides were then incubated at 37°C in the presence of 5% CO_2_ for 2 h. The neutrophils were fixed for 30 min using methanol, after the process of incubation. The gels were gently removed after fixation, and the neutrophils were stained with Giemsa stain.

The slides were then examined at a 100x magnification using a digital microscope. Motic-3.2 software was used to measure the distance traveled by the leading front of cells toward the FMLP-containing wells [40].

*(4) Nitric Oxide Scavenging Assay*. Borra and Gurumurthy explained the procedure in detail, in which a solution of 10 mM sodium nitroprusside in phosphate-buffered saline (PBS) pH 7.4 was combined with 0.5 ml of drug solutions at different concentrations ranging from 10 to 50 *μ*g/ml and ascorbic acid at concentrations of 25 to 200 *μ*g/ml. This combination was kept at a temperature of 25°C. 0.5 ml of the incubation solution was collected after 150 minutes and mixed with 0.5% of the Griess reagent, 0.5% of the sulfanilic acid reagent (0.33 percent prepared in 20% glacial acetic acid at room temperature for 5 minutes), and 0.1 percent *w*/*v* of the naphthyl ethylene diamine dihydrochloride (1.0 ml). After 30 minutes of incubation at room temperature, the mixture's absorbance at 540 nm was recorded [41].

## 3. Results and Discussion

### 3.1. Physicochemical Analysis and Preliminary Phytochemical Screening of HES

The HES pills were light olive brown and oval (solid) with a distinctive agreeable taste and astringent smell. The pills were kept in a cold, dark area in firmly covered containers, shielded from moisture, light, and temperature. Physicochemical examination found a slightly basic pH of 6.5 as stated in Tables 1 and 2.

The presence of numerous secondary metabolites like alkaloids, tannins, flavonoids, proteins, and the mucilage may explain the therapeutic benefits of HES tablets. As a result, preliminary screening assays can aid in the detection of bioactive components, which can lead to medication development and discovery. Furthermore, these tests make it easier to estimate the quantity of pharmacologically active chemical substances and to separate them qualitatively. In the HES extract, preliminary phytochemical screening with several qualitative chemical assays revealed the presence of reducing sugars, protein, amino acid, alkaloids, and tannins, whereas carbohydrates, glycosides, flavonoids, saponins, fats and oils, and steroids were lacking.

### 3.2. *In Vivo* Anti-inflammatory Activity

#### 3.2.1. Experimental Method (Carrageenan-Induced Rat Paw Edema)

In a carrageenan-induced paw edema test, rats received subplantar injections of carrageenan that displayed increased and decreased paw thickness with time. In the normal control group at *t* = 0, paw thickness was observed at 3.026 ± 0.89 cm which remained the same after 24 hrs. In the carrageenan control group, paw thickness showed an exponential increase and displayed significance at *p* < 0.001. It was 3.031 ± 0.076 cm at *t* = 0, which was increased after 24 hrs to 4.261 ± 0.123 cm. In the HES-treated group, paw thickness was 3.021 ± 0.084 at *t* = 0, but it showed an increase in paw inflammation after one hour, i.e., 3.195 ± 0.082 cm which again showed a decrease in paw thickness up to 4th hour, i.e., 3.018 ± 0.078, 2.98 ± 0.032, and 2.684 ± 0.061 at *t* = 2, 3, and 4, respectively. It showed again getting back to the normal thickness of paw at *t* = 24 hrs, i.e., 3.029 ± 0.118 cm. In diclofenac sodium-treated groups, it displayed the same pattern as demonstrated by the HES-treated group. All the results obtained were significant with the control group. The values are tabulated in Table 3 and the graph paw thickness Vs time is illustrated in Figure 1.

### 3.3. Paw Withdrawal Threshold (Von Frey Test)

#### 3.3.1. Effect of HES on Paw Withdrawal Threshold

In Figure 2 and Table 4, the Von Frey test reporting pain threshold measurement is displayed. A decreased withdrawal response was observed through a nonnoxious mechanical stimulation of the paw (allodynia-like measure) in carrageenan-treated animals, which maintained a plateau at 2 and 3 hours after treatment. Treatment with HES (*p* < 0.001) showed a significant decrease in pain from 0 to 60 min, and similar treatment with standard oxycodone also showed a significant decrease (*p* < 0.001) in pain from 0 to 60 min. Thus, HES and the standard drug showed complete blockade of carrageenan-induced hypersensitivity.

### 3.4. Acetic Acid-Induced Vascular Permeability

#### 3.4.1. The Impact of HES on Evans Blue Dye Extravasation into the Rat Peritoneal Cavity

Standard reduced the dye leakage into the peritoneum more effectively when compared to HES and control. HES has an anti-inflammatory effect because it reduces the permeability of blood vessels, which results in less dye leakage. In the present method, HES (*p* < 0.001) and metformin (*p* < 0.001) have shown significant inhibition of dye leakage (Figure 3).

#### 3.4.2. Effects of HES on Tail Withdrawal Reflexes in Rats Induced by Tail Immersion

All three samples have shown significant inhibition concerning control (HES, *p* < 0.001). From Table 5 and Figure 4, it is evident that all the formulation had shown significant analgesic activity. Dextropropoxyphene had a significantly higher concentration than this.

#### 3.4.3. Rats' Resistance to Adjuvant-Induced Arthritis after Treatment with HES

From day 8 to day 28, the AIA group's paw volume was considerably higher than that of the regular control group (*p* < 0.001). Paw edema was significantly reduced in the HES and MTX-treated groups compared to the untreated controls (*p* < 0.001) (Figure 5).

#### 3.4.4. Effect of HES on Rats Treated with Freund's Complete Adjuvant on Hematological Parameters

Arthritis-related hematological alterations are shown in Table 6 and Figure 6. Levels of WBC, platelet count, and ESR were increased in arthritic rats, while the level of RBC was decreased. These levels were observed to be near normal on treatment with standard drugs, whereas HES has shown less significant or no significance when compared to the AIA group.

### 3.5. In Vitro Models

#### 3.5.1. Determination of TAC and FRAC

The TAC and FRAC of HES are shown in Table 7. When compared to normal catechin, HES had significantly higher antioxidant activity. At the concentration of 100 *μ*g/ml, the absorbance of HES was in the range of 0.584 ± 0.053 to 1.89 ± 0.076, while at 150 *μ*g/ml, the range was 0.874 ± 0.043 to 2.394 ± 0.064. An increase in therapeutic dosage resulted in an increase in total antioxidant activity.

A moderate to high FRAC was seen in HES when drug concentrations were boosted in the animal. At 100 *μ*g/ml, the absorbance was in the range of 0.975 ± 0.056 to 3.409 ± 0.065, while at 150 *μ*g/ml, the range was 1.345 ± 0.086 to 3.225 ± 0.067. Results show that HES has the greatest TAC and FRAC values, which is similar to the catechin and ascorbic acid standards.

#### 3.5.2. Evaluation of the DPPH Radical Scavenging Activity of HES

Figure 7 and Table 8 illustrate the free radical scavenging activity of both HES and BHT. At a concentration of 100 *μ*g/ml, the scavenging activity of HES and BHT was 78 ± 0.64 and 95 ± 0.94 *μ*g/ml. By suppressing the DPPH radical with a high inhibition value, the extract demonstrated concentration-dependent antioxidant activity. The approach relies on the creation of the nonradical form DPPH-H by the reaction, which reduces the DPPH solution in the presence of a hydrogen donor antioxidant. The extract was able to convert the DPPH radical into yellow diphenyl picrylhydrazine, which was stable. Because of its propensity to contribute hydrogen, ascorbic acid has been discovered to decrease and discolor 1,1-diphenyl-2-picrylylhydrazyl. HES extract appears to be able to give hydrogen while also acting as an antioxidant. As the concentration of the extract rises, so does the effect of elimination.

### 3.6. Hydroxyl Radical Scavenging Capabilities of HES

HES has exhibited a dose-dependent hydroxyl radical scavenging activity as illustrated in Figure 8 and tabulated Table 9. The scavenging activity of HES at a concentration of 100 *μ*g/ml was 47 ± 0.75, while that of catechin was 63 ± 0.84 *μ*g/ml.

### 3.7. *In Vitro* Activity of HES on Human PMN Cell

In an agarose experiment of PMN cell chemotaxis, the drugs stimulated the migration of PMN cells toward the chemoattractant FMLP. According to Figure 9, all groups' stimulation of PMN cell chemotaxis (measured in micrometres) was significant (HES *p* < 0.001).

### 3.8. Nitric Oxide Scavenging Assay

In tests, the formulation had just a little ability to reduce levels of nitric oxide (NO). Drug concentration raises the percentage of inhibition. After 150 minutes of incubation at 25°C with sodium nitroprusside solutions in PBS, NO production was detected. As shown in Table 10, the IC_50_ for HES was 41.59 ± 2.45 *μ*g/ml, while the IC_50_ for ascorbic acid was 186.34 ± 3.28 *μ*g/ml.

## 4. Conclusion

One of the most frequently prescribed Unani formulations for the treatment of inflammation and arthritis is Habb-e-Suranjan. In the present investigation, we tried a scientific attempt to evaluate its anti-inflammatory potential using different *in vitro* and *in vivo* models. A battery of tests evaluating a range of activities such as carrageenan-induced rat paw edema, Von Frey test, adjuvant-induced arthritis (AIA) in rats, hydroxyl radical scavenging activity test, nitric oxide scavenging activity test, free radical scavenger DPPH, and *in vivo* and *in vitro* anti-inflammatory activities have been demonstrated. The inclusion of diverse polyherbal components, which is a recognized powerful antioxidant and anti-inflammatory, could explain Habb-e-Suranjan's effectiveness. Overall, the current study shows the anti-inflammatory and antioxidant ability of formulation, which not only rationalizes some ethnomedicinal claims but also identifies a promising candidate for further research, particularly in chronic inflammatory disorders like rheumatoid arthritis. More study is needed to be done to find the biomolecules that are responsible for the anti-inflammatory and antioxidant effects. In the future, we are aiming to investigate its effectiveness using more quality *in vivo* models and by estimating more precise biochemical parameters followed by histological examination.

## Figures and Tables

**Figure 1:** Paw edema caused by carrageenan treatment with HES.

**Figure 2:** Effect of HES on paw withdrawal threshold.

**Figure 3:** The impact of HES on Evans Blue dye extravasation into the rat peritoneal cavity.

**Figure 4:** Tail withdrawal reflexes elicited by the tail immersion technique in rats are affected by HES.

**Figure 5:** In rats, HES has an anti-inflammatory impact on AIA.

**Figure 6:** The hematological parameters of rats treated with Freund's complete adjuvant and the effect of HES on these parameters.

**Figure 7:** Evaluation of the DPPH radical scavenging activity of HES.

**Figure 8:** Hydroxyl radical scavenging capabilities of HES and CA.

**Figure 9:** Effect of HES on FMLP-induced chemotaxis of PMN cells. Values are expressed as mean ± SEM. ^a^*p* < 0.001 when compared to the control group.

**Table 1:** Organoleptic character.

Sr. no.	Parameters	Observation
1	Size	Oval
2	Color	Light olive brown
3	Taste	Agreeable
4	Odor	Astringent
5	Appearance	Habb (pills)

**Table 2:** Physiochemical character.

Sr. no.	Parameters	HES
1	Friability test	0.83%
2	Hardness test	5.5 kg/cm^2^ (Monsanto)
3	Weight variation	0.112
4	Disintegration time	32 min
5	A pH of 1% solution	6.5
6	10% solution	5.6

**Table 3:** Effect of HES on carrageenan-induced paw edema.

Treatment	Paw thickness of rats (cm)					
	0 hr	1 hr	2 hr	3 hr	4 hr	24 hrs
Group I: normal control	3.026 ± 0.89	3.026 ± 0.073	3.026 ± 0.082	3.026 ± 0.092	3.026 ± 0.074	3.026 ± 0.109
Group II: carrageenan control	3.031 ± 0.076	3.189 ± 0.069	3.392 ± 0.087	3.628 ± 0.093	3.732 ± 0.061	4.261 ± 0.123
Group III: HES	3.021 ± 0.084^∗∗∗^	3.195 ± 0.082^∗∗∗^	3.018 ± 0.078^∗∗∗^	2.98 ± 0.032^∗∗∗^	2.684 ± 0.061^∗∗∗^	3.029 ± 0.118^∗∗∗^
Group IV: diclofenac sodium (standard)	3.035 ± 0.086^∗∗∗^	3.098 ± 0.087^∗∗∗^	2.961 ± 0.069^∗∗∗^	2.92 ± 0.077^∗∗∗^	2.899 ± 0.088^∗∗∗^	3.034 ± 0.139^∗∗∗^

Values are expressed as mean ± SEM. ^∗^*p* < 0.001 compared to control group and ^∗∗∗^*p* < 0.001 compared to carrageenan control group.

**Table 4:** Effect of HES on paw withdrawal threshold.

Treatment	Paw withdrawal threshold (g)				
	0 min	15 min	30 min	45 min	60 min
Normal control	0.64 ± 0.02	0.65 ± 0.02	0.67 ± 0.02	0.69 ± 0.02	0.66 ± 0.02
Carrageenan control	0.29 ± 0.01	0.23 ± 0.03*^α^*	0.26 ± 0.03*^α^*	0.27 ± 0.02*^α^*	0.26 ± 0.02*^α^*
HES	0.31 ± 0.03	0.51 ± 0.02^a^	0.63 ± 0.02^a^	0.53 ± 0.03^a^	0.50 ± 0.03^a^
Standard	0.38 ± 0.02	0.81 ± 0.01^a^	0.85 ± 0.01^a^	0.83 ± 0.01^a^	0.79 ± 0.02^a^

Values are expressed as mean ± SEM. *^α^p* < 0.001 compared to control group and ^a^*p* < 0.001 compared to carrageenan control group.

**Table 5:** Tail withdrawal reflexes elicited by the tail immersion technique in rats are affected by HES.

Drug (dose)	Before treatment (sec)	After treatment (sec)
Control (saline)	5.7 ± 0.082	5.8 ± 0.099
HES (100 mg/kg)	6.0 ± 0.053	7.3 ± 0.19^a^
Dextropropoxyphene (65 mg/kg)	5.7 ± 0.066	10 ± 0.16^a^

**Table 6:** The hematological parameters of rats treated with Freund's complete adjuvant and the effect of HES on these parameters.

Group	WBC count (10^3^/mm^3^)	RBC (× 10^6^/*μ*l)	Platelet count (10^5^/mm^3^)	ESR (mm/hr)
Normal control	8.7 ± 0.25	6.0 ± 0.15	2.4 ± 0.16	3.7 ± 0.19
AIA control	12 ± 0.31*^α^*	4.3 ± 0.28*^α^*	3.5 ± 0.11*^α^*	5.6 ± 0.15*^α^*
HES	10 ± 0.34^b^	5.5 ± 0.18^c^	2.9 ± 0.07^c^	5.2 ± 0.16
Standard	9.5 ± 0.26^a^	6.0 ± 0.21^a^	2.5 ± 0.12^a^	4.4 ± 0.09^c^

**Table 7:** Absorbance HES at two different concentrations.

Drugs	TAC		FRAC	
	At 100 *μ*g/ml	At 150 *μ*g/ml	At 100 *μ*g/ml	At 150 *μ*g/ml
HES	0.934 ± 0.098	1.284 ± 0.095	1.576 ± 0.032	1.874 ± 0.056
CA	1.89 ± 0.076	2.394 ± 0.064	—	—
AA	—	—	3.409 ± 0.065	3.225 ± 0.067

CA: catechin; AA: ascorbic acid. *n* = 3, mean ± SD.

**Table 8:** Evaluation of the DPPH radical scavenging activity of HES.

Concentration (*μ*g/ml)	BHT	HES
0	0	0
12.5	80	43
25	93	50
50	95	59
100	95	78
150	95	83

**Table 9:** Hydroxyl radical scavenging capabilities of HES and CA.

Concentration (*μ*g/ml)	CA	HES
0	0	0
12.5	16	24
25	22	34
50	37	40
100	63	47
150	84	51

**Table 10:** IC_50_ value for *in vitro* nitric acid scavenging activity.

Sr. no.	Sample	Nitric oxide (*μ*g/ml)
1	HES	41.59 ± 2.45
2	Ascorbic acid	186.34 ± 3.28

## Data Availability

The data used to support the findings of this study are included within the article.
